# Development Strategy of Intelligent Digital Library without Human Service in the Era of “Internet +”

**DOI:** 10.1155/2022/7892738

**Published:** 2022-10-10

**Authors:** Hongmei Wang, Jian Ding

**Affiliations:** ^1^Northeast Forestry University, Library, Harbin 150040, China; ^2^Harbin Conservatory of Music, Harbin 150028, China; ^3^Postdoctoral Program of Heilongjiang Hengxun Technology Co., Ltd., Harbin 150090, China

## Abstract

Internet technology has a great impact on the application and development of libraries. In order to provide users with more convenient and efficient services, this paper puts forward the development strategy of unmanned intelligent digital libraries in the era of “Internet +.” Design by IntelliSense module, network transmission module, data storage and analysis module, and intelligent service module of no wisdom digital library service mode, IntelliSense module using RFID technology, close range wireless communication technology, and other Internet technologies to collect the wisdom of unmanned services of all kinds of information in the digital library; use network transmission module of the wireless LAN network, Internet technology such as RFID network to transmit information collected to store in a data storage and analysis module; and at the same time using *k*-means clustering algorithm in data mining techniques such as analysis of collected data, based on the analysis results provide users with intelligence services such as search, wisdom is recommended. The experimental results show that the developed strategy meets the expected functional requirements, can accurately perceive the location of data, and effectively realize the intelligent service function.

## 1. Introduction

Under the background of the Internet era, compared with previous libraries, the system service of smart digital libraries is becoming more and more perfect, and the information behavior of users presents the characteristics of the Internet [1]. Users' access to information has taken on a new form and is constantly developing in the direction of intelligence, informatization, digitization, and modernization [2], and information behavior is becoming more and more convenient. In the “Internet +” era, information resources are more abundant and platform systems are more integrated. However, at present, there are some problems in the service of a smart digital library, which need to be handled in time, establish and improve the mechanism, and improve the service quality of the smart digital library. “Internet +” brings a new development opportunity for the construction of a smart digital library. Combined with the construction of a smart digital library, it can use “Internet +” to fuse different information [3], cross-border integrate information, and achieve the goal of information service. “Internet +” is the product of social development and the crystallization of science, technology, and economic development [4]. The construction of the smart digital library is affected by the Internet. It combines other industries with library information so that library information can be combined with all industries and fields that can be connected and contact institutions in different places.

The concept of a smart digital library was first put forward by foreign library circles [5]. Whether it is theoretical research or practical research, its starting point and purpose are to realize the universality and intelligence of a smart digital library, so as to provide users with intelligent and personalized services. Around 2003, the library of University of Oulu in Finland launched a service called “smart library” [6]. Smart library is a space-free and perceptible mobile library service that can be used anywhere there is Internet. As for the definition of a smart digital library, different scholars in China have given different expressions from different angles. From the perspective of sensor computing, Yan Dong proposed that smart digital library = library + Internet of Things + cloud computing + intelligent equipment [7]; from the perspective of big data and ubiquitous learning, Wang Weiqiu proposed that smart digital library was the integration of digital library, intelligent perception equipment, big data analysis, and ubiquitous learning space [8]; from the perspective of humanized service and management, Pingping proposed that the smart digital library had changed the interaction mode between users and library facilities, systems and information resources through modern information technology, so as to make the service and management of the library more intelligent [9]. Based on the views of the abovementioned scholars, it can be considered that the smart digital library should be a new generation library that takes the digitization of resources as the premise and is based on the Internet of Things technology, Internet technology, and mobile terminals, guided by the needs of readers, is not limited by space, can be perceived, and continuously improves the reader experience, which is the future development direction of the library.

In recent years, with the continuous development of ubiquitous Internet technology based on mobile Internet and Internet of Things and the continuous expansion of mobile terminal functions, the information service mode based on situational perception, ubiquitous computing, intelligent judgment, and multidimensional interaction will be the main direction of the development of smart library in the future. At present, some scholars have done relevant research on the development strategy of a smart digital library. Wu introduced the intelligent library personalized recommendation service system based on intelligent technology [10]; combined with the characteristics of a ubiquitous and intelligent smart library, Bi et al. constructed a hierarchical model of a ubiquitous smart library from the bottom-up from the perspective of user service [11]; and Cui and Wu introduced the intelligent service system of Library of Nanjing University, including the construction and transformation of physical venues, the construction of information service platform and the construction of intelligent services, and introduced the construction and implementation of its intelligent library in detail [12, 13].

In order to predict the future development of the unmanned service command digital library, this paper studies the development strategy of the unmanned service smart digital library in the era of “Internet +,” and provides users with smart search, smart recommendation, and other smart services, hoping that the research content can improve the service quality of the smart digital library.

## 2. Materials and Methods

“Internet +” refers to a new form of business developed by the Internet under the impetus of innovation 2.0, and a new form of economic and social development evolved and spawned by the Internet under the impetus of knowledge society innovation 2.0. “Internet +” is a further practical achievement of Internet thinking. It represents an advanced productive force, promotes the continuous evolution of economic forms, drives the vitality of social and economic entities, and provides a broad network platform for the reform, innovation, and development of unmanned smart digital libraries.

### 2.1. Resource Feature Extraction of Unmanned Intelligent Digital Library

The intelligent service mode of an unmanned intelligent digital library is composed of four main parts: intelligent sensing module, network transmission module, data storage and analysis module, and intelligent service module, as shown in Figure 1.

Intelligent sensing module refers to the use of a variety of Internet technologies to connect users, information resources, unmanned intelligent digital libraries, and so on so that they become an organic whole, so as to achieve the interconnection of information among the three.

When extracting the resource features of the unmanned service intelligent digital library, it is regarded as the combination of the user's interests and the resource characteristics, that is, the matching of the student's personalized portrait and the resource features of the unmanned service intelligent digital library. Therefore, after completing the construction of the personalized portrait of students, the resource features of the unmanned intelligent digital library are extracted [8]. Then the matching calculation is carried out for the attribute characteristics of the resources of the unmanned intelligent digital library, and the conditions are provided for the subsequent resource recommendation and detailed display. In the specific operation, it is necessary to determine the distribution of resource data of the unmanned intelligent digital library. In the heterogeneous data storage environment of the unmanned intelligent digital library, the decision-making feature preference of resource data is introduced, and the integration of student personalized portrait and resource feature data is realized. In this process, the following formula can be used:

(1) $$\begin{array}{c} W_{abc}=\frac{A_{a}}{\underset{i=1}{\sum }\left(B_{i}-C_{i}\right)}\text{.} \end{array}$$

In Equation (1), *W*_*abc*_ represents the resource characteristic data of the unmanned intelligent digital library obtained through the abovementioned operation; *A*_*a*_ represents a user personalized portrait tag corresponding to the feature data; *B*_*i*_ represents the characteristic value of all unmanned smart digital library resources; *C*_*i*_ represents the personalized portrait label of the student corresponding to a specific unmanned intelligent digital library resource. According to the abovementioned equation, complete the fusion of student personalized portrait and resource feature data, and then need to fuse all resource feature data. The specific equation is given as follows:

(2) $$\begin{array}{c} G_{H}=K_{L}\times K_{J}\times W_{abc}. \end{array}$$

In Equation (2), *G*_*H*_ represents the objective function of resource feature extraction of unmanned intelligent digital library; *K*_*J*_ represents the weight coefficient during feature extraction under a certain recommended delay *J* condition; and *K*_*L*_ represents the feature extraction weight when the consumption is *L* in the feature extraction of the resources of an unmanned intelligent digital library. According to the abovementioned operations, the integration of various resources in the unmanned intelligent digital library is realized. After the integration, the feature data needs to be reconstructed in multidimensions. The fusion matching method can be introduced to reconstruct the data, and the reconstructed data can be imported into the recommendation database of the unmanned intelligent digital library according to the abovementioned operation, so as to complete the resource feature extraction task of the entire digital unmanned intelligent digital library.

### 2.2. RFID-Based Book Location Sensing Algorithm

FRID technology is used to collect book locations in an intelligent digital library without human service. According to the workflow of FRID technology, the sensing method based on frequency domain phase difference is used to sense the distance between tag reader and tag in the two-dimensional space of an intelligent digital library without human service; based on the two-dimensional spatial distance sensing results of the intelligent digital library without human service, the trilateral measurement method is selected to sense the three-dimensional coordinate position data of the book tag to be perceived in the intelligent digital library without human service.

#### 2.2.1. Two-Dimensional Distance Perception

According to the working process of FRID technology, the reader transmits carrier signals with different frequencies [14–16]. After a certain distance, the signal is received and reflected by the book tag. The reader obtains the reflected signal and determines the distance between the book target (the tag to be perceived) and the tag reader (the location coordinates are known) based on the signal phase difference. The specific process is given as follows.

Ignoring the time required for the process from book tag receiving to transmitting carrier signal, Δ*s* and *a* are respectively used to represent the time required for the process from reader transmitting carrier signal to receiving reflected signal and the propagation speed of RF signal in the air, so as to obtain the expression of speed distance *d*:

(3) $$\begin{array}{c} d=a\Delta s\text{,} \end{array}$$

*where* *β* and *p* are respectively represented the phase and carrier frequency experienced by the reader carrier signal from the transmission to reception.

#### 2.2.2. 3D Position Perception

After determining the distance between the book tag to be perceived and the tag reader in the two-dimensional space of the intelligent digital library without human service, it can select the trilateral measurement method to perceive the three-dimensional coordinate position data of the book tag to be perceived in the intelligent digital library without human service [17].

*d*_*i*_(*i*=1,2,3) represents the distance between the three readers and the tag, and the coordinate (*x*_*i*_, *y*_*i*_)(*i*=1,2,3) of each reader is known, so as to obtain

(4) $$\begin{array}{c} d_{i}=\sqrt{{\left[\left(x_{i}-x_{0}\right)+\left(y_{i}-y_{0}\right)\right]}^{2}.} \end{array}$$

On this basis, the position coordinate (*x*_0_, *y*_0_) of the book tag to be perceived in the intelligent digital library without human service can be determined by constructing the equation.

The distance relationship between the reader *i* and the book tag to be perceived in the three-dimensional space of the intelligent digital library without human service can be described by the following equation:

(5) $$\begin{array}{c} d_{i}^{2}={\left[\left(x-x_{i}\right)+\left(y-y_{i}\right)+\left(z-z_{i}\right)\right]}^{2}\text{.} \end{array}$$

Equation (5) is defined as a spherical equation. Since the tag is a common point, according to the geometric relationship, the position data of the book tag to be perceived in the intelligent digital library without human service determined by four readers [18] can be obtained, so as to obtain the distance equation group between the book tag and the reader.

From the abovementioned description, it can be seen that accurately obtaining the distance between the book tag to be perceived and the tag reader in the two-dimensional space of the intelligent digital library without human service is the basis for obtaining the high-precision three-dimensional position coordinate data of the books in the intelligent digital library without human service.

If the distance between each tag reader and the book tag has high accuracy, and the tag reader is set in different corners of the intelligent digital library without human service, which can avoid multiple tag readers from being in the same straight line with the book tag, then Equation (5) must have a unique solution. However, in the process of actually perceiving the book located in the intelligent digital library without human service, the calculation result of the distance between the tag reader and the book tag has a certain error [19], resulting in no solution in Equation (5). In order to solve this problem, it is necessary to use the selected gradient descent method to calculate the solution that makes Equation (5) approximate.

A coordinate position of the book tag to be perceived in the environment of the intelligent digital library without human service is selected, and Equation (6) is used to determine the distance between each reader and the coordinate point of the book to be perceived as follows:

(6) $$\begin{array}{c} d_{0i}=\sqrt{{\left[\left(x_{0}-x_{i}\right)+\left(y_{0}-y_{i}\right)+\left(z_{0}-z_{i}\right)\right]}^{2}}\text{.} \end{array}$$

The actual distances *d*_*i*_ and *d*_0*i*_ between the book tag and the *i*th reader are subtracted to obtain the error *w*_0*i*_.

After perceiving the relevant information of the intelligent digital library without human service, it can use the network transmission module to transmit the perceived data to the data storage and analysis module and store it. Data mining technology is used to analyze the perceived data, and realize different smart services according to the analysis results.

### 2.3. Data Storage Analysis of Intelligent Digital Library without Human Service Based on Data Mining

Based on the perceived data information of the intelligent digital library without human service, a personalized service-oriented big data mining process of the intelligent digital library without human service is designed, as shown in Figure 2.

According to Figure 2, data mining, also known as knowledge discovery in the database, is a hot topic in the field of artificial intelligence and database research. It helps decision-makers adjust market strategies, reduce risks and make correct decisions. In the big data mining implementation scheme shown in Figure 2, the main modules are divided into data collection, role modeling, algorithm implementation and result storage, and front-end application. Role modeling, algorithm implementation, and result storage belong to the offline part, and the online part involves data collection and front-end application [20].

#### 2.3.1. K-Means Clustering Algorithm

The clustering algorithms in the process of data analysis stored in the intelligent digital library without human service mainly include hierarchy-based, partition-based, and density-based algorithms [21], among which the most commonly used and effective is the partition-based K-means clustering algorithm. Its specific implementation process is given as follows:

1. Firstly, randomly select *k* vectors as the center of each class.
2. Let *E* be a two-dimensional membership matrix of *c* × *n*. If the *j*-th vector *x*_*j*_ belongs to class *i*, the element *e*_*ij*_ in matrix *E* is 1, otherwise, it is 0. That is, for each *k* ≠ *j* and when ‖*X*_*j*_ − *C*_*i*_‖ ≤ ‖*X*_*j*_ − *C*_*k*_‖, *e*_*ij*_ value is 1, otherwise the value of *e*_*ij*_ is 0.
3. Calculate the value of objective function *J* according to *e*_*ij*_, and stop if it is less than a threshold or the difference between two consecutive times is less than a threshold.
4. Calculate the center *C*_*i*_ of each cluster *G*_*i*_ according to *e*_*ij*_: $C_{i}=\underset{i\in G_{j}}{\sum }X_{i}/\left|G_{i}\right|$, and *G*_*i*_ is the number of elements in the cluster. Then go back to step (2).

Although K-means algorithm has attracted much attention due to its advantages such as simplicity and efficiency, it still has some limitations, mainly as follows:

1. Clustering results are excessively dependent on the selection of initial values [22], and the accuracy and stability of clustering results are poor
2. The algorithm is very sensitive to outliers [23], and there are large errors in the clustering results

#### 2.3.2. Improved K-Means Algorithm

To solve the abovementioned problems, an improved K-means algorithm based on the principle of natural nearest neighbor density and maximum-minimum distance is proposed to optimize the selection of initial clustering centers. Starting from the internal distribution characteristics of the stored data in the intelligent digital library without human service [24], the algorithm can adaptively determine the data density, avoid the problem of artificial parameter setting, and objectively and truly reflect the distribution characteristics of the stored data in the intelligent digital library without human service, so as to find a high-quality initial center to solve the disadvantage that the initial center point randomly selected by the traditional K-means algorithm is not representative. At the same time, it can eliminate the influence of outliers on the clustering results, so as to improve the accuracy and effectiveness of the final analysis results when clustering the relevant data of the intelligent digital library without human service. The improved algorithm flow is given as follows.

**Step 1 .**

For the relevant data set of the intelligent digital library without human service, find out the natural nearest neighbor of the relevant data sample point *x*_*i*_ of each intelligent digital library without human service according to the natural nearest neighbor search algorithm, and determine the density function of the relevant data points of each intelligent digital library without human service. The equation is given as follows:

(7) $$\begin{array}{c} d_{e}\left(x_{i}\right)=\frac{1}{\underset{x_{j}\in NN_{nb\left(i\right)}\left(i\right)}{\sum }k_{i}\left(x_{i},x_{j}\right)}\times n_{b}\left(i\right)\text{.} \end{array}$$

In Equation (7), *n*_*b*_(*i*) represents the number of times that the relevant data sample points of the intelligent digital library without human service appear in the *r* neighborhood of the relevant data sample objects of the other unserviceable smart digital libraries, that is, the number of natural nearest neighbors of sample *i*, *NN*_*nb*(*i*)_(*i*) represents the natural nearest neighbor set of the relevant data points of each intelligent digital library without human service, and *k*_*i*_(*x*_*i*_, *x*_*j*_) is the European distance between the relevant data points *x*_*i*_ and *x*_*j*_ of the intelligent digital library without human service.

**Step 2 .**

Delete the relevant data sample points of sparse intelligent digital library without human service satisfying condition to obtain the relevant data intensive sample point set *X*′ of an intelligent digital library without human service.

**Step 3 .**

Select the highest density in *X*′, i.e., *x* of *de* *ns*_max_(*x*), as the first initial clustering center *c*_1_; the longest distance mentioned above is the standard [25], to look for the second center point *c*_2_; and so on until we get *k* initial clustering centers *C*={*c*_1_, *c*_2_, ⋯, *c*_*k*_}.

**Step 4 .**

Calculate the attribute weight of the dataset.

**Step 5 .**

Calculate the weighted Euclidean distance between all the relevant data sample points of the intelligent digital library without human service and the *k* initial cluster centers obtained in step 3, where *x* ∈ *X* and *c* ∈ *C*. Assign each relevant data point of the intelligent digital library without human service to the nearest center [26], forming *k* clusters, and each cluster is represented by its cluster center.

**Step 6 .**

Recalculate the cluster center according to the clustering results of step 5.

**Step 7 .**

Repeat step 5 with the results in step 6 as input until the cluster center does not change or the cluster reaches the maximum number of iterations.

**Step 8 .**

Output *k* class clusters.

It can be achieved through the abovementioned process.

## 3. Experimental Results

This paper studies the development strategy of the intelligent digital library without human service in the “Internet +” era. Taking the University Library as the research object, this paper adopts the development strategy to build an intelligent digital library without human service and verifies the actual performance of the development strategy studied in this paper through experiments. The results are given as follows.

### 3.1. Functional Test

The main content of the functional test is to test the performance of book borrowing and automatic return under the development strategy studied in this paper. In order to ensure the robustness of book borrowing and automatic book return to the input content, the black box test method is adopted based on the functional requirements of different module designs.

#### 3.1.1. Performance Test of Book Borrowing

The black box test method is used to test the book borrowing function under the development strategy of this paper. The test cases, expected outputs, and actual outputs are shown in Table 1.

According to the analysis of Table 1, under the development strategy of this paper, book borrowing first needs to scan the user's library card to determine the user's identity. After determining the identity of the book borrower, it needs to scan the books to bind the relevant information of the book borrower (library card number) and book information (ISBN number), and then click the OK button to complete the book borrowing. According to the analysis of Table 1, the book borrowing function under the development strategy of this paper can identify whether the user's relevant information (library card number) is registered or not, judge the upper limit of books that can be borrowed according to the user's relevant information (library card number), and prompt “user does not exist” for unregistered users.

The actual output of the relevant test cases in Table 1 is completely consistent with the expected output, which shows that the book borrowing function under the development strategy of this paper meets the expected requirements.

#### 3.1.2. Performance Test of the Automatic Book Return Module

The black box test method is used to test the automatic book return function of the research object under the development strategy of this paper. The test cases, expected outputs, and actual outputs are shown in Table 2.

Analysis of Table 2 shows that the automatic book return function under the development strategy of this paper can identify whether the books exist, whether they are borrowed, whether they are returned, and the location of the returned books. The actual output of the relevant test cases in Table 2 is completely consistent with the expected output, which shows that the design of the automatic book return function under the development strategy of this paper meets the expected requirements.

### 3.2. Position Perception Error Analysis

Select different types of books (poetry books, astronomy books, and medical books) and analyze the perception results of book sample location data under the development strategy of this paper. The results are shown in Figures 3–5.

From Figure 3 to Figure 5, under the development strategy of this paper, the position perception error of different types of book samples in different directions is controlled within 4.5 cm, which is significantly lower than the standard position perception error threshold of 10 cm generally recognized in relevant fields. The reason is that this method designs a personalized service-oriented big data mining process for unattended smart digital libraries based on the perceived data information of unattended smart digital libraries, which is conducive to controlling errors to a certain extent. This shows that under the development strategy of this paper, the position perception accuracy of different types of book samples is higher.

### 3.3. Data Mining Performance Analysis

Taking the user information in the research object as an example, according to the cluster center obtained from the clustering results, the medical book users are divided into five interest groups, and the clustering accuracy under different K values is analyzed. The results are shown in Figure 6, the specific situation of clustering division is shown in Figure 7, and the book recommendation is realized according to the user clustering results, and results are shown in Figure 8.

According to the analysis of Figure 6, under the conditions of different K values, the clustering accuracy of the method in this paper shows a trend of gradually increasing at first and then significantly decreasing. When the K value is increased from 3 to 8, the clustering accuracy of this method is improved from 93.5% to 98.5%; with the continuous improvement of K value, the clustering accuracy of this method gradually decreases. When the K value reaches 12, the clustering accuracy of this method will be less than 90%. This shows that the optimal clustering accuracy can be obtained when the K value in this method is 8.

After the user's interest group division results shown in Figure 7 are obtained, the borrowing record data of “Tonghao” users in the interest group can be analyzed as part of the reference basis for recommendation in the next step. For example, for target user 07, who likes traditional Chinese medicine, find out the most similar users in the interest group (user 33 and user 48), And recommend the relevant borrowing of these users to the user (see Figure 8). According to the analysis of Figure 8, most of the data borrowed by users 33 and 48 are borrowed by user 07, which shows that this method can effectively realize the intelligent recommendation function.

## 4. Recommendations

In view of the current development status of China's intelligent digital library without human service, this paper puts forward the following suggestions for the development of intelligent digital libraries without human service.

### 4.1. Strengthening Top-Level Design and Formulating the Action Plan of “Internet + Library”

“Internet +” has become a new engine to promote social, economic, and cultural development. The state council, provinces and cities, and industries have successively formulated “Internet +” action plans. “Internet +” also has a profound impact on libraries and promotes the transformation and development of libraries. Libraries should seize the opportunity, strengthen top-level design, scientifically formulate the “Internet + library” action plan, clarify the objectives, paths, and key measures of library transformation under the “Internet +” background, explore the implementation scheme of the “Internet + library” action plan and accelerate the deep integration of the Internet and libraries; it should strive to explore the impact of “Internet +” on library service concept, service mode, resources, organization, management, etc., have the courage to break down various obstacles incompatible with the development of “Internet +,” speed up the reform process, stimulate innovation vitality, and improve service efficiency and efficiency. In this regard, Zhejiang Provincial Public Library is at the forefront of national libraries. In July 2015, Zhejiang Library, together with 11 municipal public libraries in the province, jointly released the “Internet +” action plan of Zhejiang Public Libraries, proposing to make library services more accessible through cross-border integration, make resources easier to find, enrich resource supply, and enable the public to enjoy more fair, efficient, high-quality and convenient public cultural services.

### 4.2. Establishing and Improving the System and Articles of Association to Ensure the Storage Security of Digital Information Resources

In order to improve the service quality of digital library and ensure the effectiveness of information resources, colleges and universities need to constantly update the mechanism and concept, do a good job in the resource management and development of digital libraries, give full play to the role and value of digital library, and realize the goal of scientific management of digital library. In order to improve the service quality and order of digital library, during the construction of the university library, it is necessary to build an information resource service system, based on the interaction of administration, economy and law, give full play to the advantages of administrative and economic means, and give full play to the role of the legal system, so as to fully implement administrative, economic and legal standards, establish and improve systems and mechanisms, and form a service system for rational use and efficient management of information resources.

At the same time, it is necessary to do a good job in the management of professional equipment and computer equipment. In order to maintain and test the security of digital library in time and ensure the security and efficiency of electronic resources and network information, we should give full play to our own advantages, strengthen the management of electronic equipment and computer equipment, build and optimize the rules and regulations system so that it can have a legal basis. In the library service of colleges and universities, only by doing a good job in the management planning of digital literature and information resources can the computer application level be improved, the digital and information resources can be stored safely for a long time, the utilization and development of information resources can be done well, and the scientific and technological achievements can be fully combined with social development so that the library service of colleges and universities can develop toward the direction of digital society and actively adapt to the digital era.

### 4.3. Making a Good Job in the Construction of Service Content

The digital library of colleges and universities has the characteristics of ubiquity and digitization. College teachers and students can obtain information for the first time in different environments and at different times. In order to ensure the scientificity and rationality of information construction, it is necessary to do a good job in the construction of information resource service content.

#### 4.3.1. Providing Information Independently

This is an intelligent service mode. The service effect of information resources is good, and college teachers and students are in a passive receiving state. To predict the information of college teachers and students, it can analyze the topics of interest, analyze the information needs of college teachers and students and the contact and rules of information resources, and push the content of interest for college teachers and students, so as to provide information independently, mainly in the form of information push and data mining.

#### 4.3.2. Transmitting Information Automatically

This information resource transmission mode focuses on the system construction mode. In the system construction, the intelligent construction function is added to achieve the goal of personalized service. After university teachers and students give keywords, intellectualization can respond in time, and provide a large amount of information resources and effective product information for university teachers and students after inquiry, sorting, collection, and arrangement. Information transmission is the main form of information automation. It increases the timeliness of information interaction and reflects the advantages of digital technology and information technology.

### 4.4. Increase Expenditure and Make a Good Job in Team Building

1. Colleges and universities should do a good job in software and hardware construction, improve the expenditure on software and hardware, adjust and optimize the collection structure of the digital library, and reasonably divide the comparison between e-books and paper books. It also needs to reduce paper financial expenditure, give full play to the advantages of network resources, and increase the storage of e-book resources. During the construction of the digital library, it is gradually transitioning from traditional library construction to digital library construction, to formulate a reasonable system and planning scheme, and constantly adjust the collection policy, information purchase, literature planning, and other work. In the document collection scheme and planning, we should improve the collection of electronic information text and increase the financial expenditure on electronic document information, so that the electronic document information resources occupy a large proportion in the library, which is conducive to the development of comprehensive digital library services.
2. Do a good job in team building. Paying more attention to the construction of a talented team is conducive to the realization of personalized and professional services of University Digital Library. It should introduce professional and technical personnel and management talents, realize technical and orderly management and improve the professionalism and gradient of talent structure. As for the digital library, it is different from the previous libraries. It does not need a large area of space, does not need to build a large number of reading rooms, changes the previous paper reading form, and realizes the goal of electronic reading. Therefore, colleges and universities can transfer the network resource information and digital information collected by the library itself, or act as the supporter and guides of the network resources of the digital library, and use guidance and training to make readers increase their ability to obtain network resources and improve the ability to obtain digital information resources. In detail, colleges and universities need to enrich the level of talents, educate and train librarians in network technology and digital technology, enhance the quality of librarians, establish a reward and punishment system, employ advanced technicians, and give full play to the maximum service goal of a digital library.

## 5. Conclusion

This paper studies the development strategy of unmanned intelligent digital libraries in the era of “Internet +” and draws the following conclusions:

1. The book borrowing function under the development strategy of this paper can identify whether the relevant information of users has been registered.
2. The actual output under the development strategy in this paper is completely consistent with the expected output, indicating that the automatic return function design under the development strategy in this paper meets the expected requirements.
3. The position sensing errors of different types of book samples in different directions are controlled within 4.5 cm, and the accuracy of position sensing is high.
4. The proposed method can obtain the optimal clustering accuracy and effectively realize the intelligent recommendation function, with strong practical application performance and more convenient and efficient service for users.

## Figures and Tables

**Figure 1:** Intelligent service mode of unmanned digital library.

**Figure 2:** Implementation process of data mining.

**Figure 3:** Poetry books.

**Figure 4:** Astronomical books.

**Figure 5:** Medical books.

**Figure 6:** Clustering accuracy under different K values.

**Figure 7:** Clustering results.

**Figure 8:** Recommended results (a) User 07. (b) User 33. (c) User 48.

**Table 1:** Test cases and output of book borrowing function.

Test case ID	Expected output	Actual output
1	Please scan books	Please scan books
2	Please scan the library card	Please scan the library card
3	Wrong library card number input	Wrong library card number input
4	Exceeding the maximum borrowing amount	Exceeding the maximum borrowing amount
5	Borrowing succeeded	Borrowing succeeded

**Table 2:** Test cases and output of automatic book return module.

Test case ID	Expected output	Actual output
1	Return the book successfully	Return the book successfully
2	The ISBN number of this book does not exist	The ISBN number of this book does not exist
3	Please scan books	Please scan books
4	The book has been returned	The book has been returned
5	This book is placed in column X of XX cabinet in XX district	This book is placed in column X of XX cabinet in XX district

## Data Availability

The raw data supporting the conclusions of this article will be made available by the authors, without undue reservation.
